RETRACTED

# Effects of Comprehensive Nursing Based on Orem's Self-Care Theory on Symptom Improvement and Pregnancy Outcome in Patients with Antiphospholipid Syndrome: A Retrospective Cohort Study

**DOI:** 10.1155/2022/4133812

**Published:** 2022-05-19

**Authors:** Meng Bi, Lingyuan Meng, Liying Bai

**Affiliations:** Obstetrics Department of Beijing Chaoyang Hospital, Capital Medical University 100020, China

## Abstract

**Objective:**

A retrospective cohort study was conducted to explore the effects of comprehensive nursing based on Orem's self-care theory on symptom improvement and pregnancy outcomes in patients with antiphospholipid syndrome (APS).

**Methods:**

Sixty patients with antiphospholipid antibody syndrome treated in our hospital from February 2019 to April 2021 were enrolled. The control group received comprehensive nursing, while the study group received comprehensive nursing based on Orem's self-care theory. Nursing satisfaction, self-nursing ability, anxiety score, social support status, pregnancy outcome, and the score of life quality were compared between the two groups.

**Results:**

First of all, we compared the nursing satisfaction, the study group was very satisfied in 23 cases, satisfactory in 5 cases, general in 2 cases, the satisfaction rate was 100.00%. While in the control group, 11 cases were very satisfied, 10 cases were satisfied, 4 cases were general, and 5 cases were dissatisfied, the satisfaction rate was 83.33%. The nursing satisfaction in the study group was higher compared to the control group (*P* < 0.05). Secondly, the self-concept, sense of self-care responsibility, self-nursing skills, health knowledge, and total score of the study group were higher compared to the control group (*P* < 0.05). After intervention, the anxiety scores of the two groups decreased. Compared between the two groups, the anxiety scores of the study group before intervention and 1 week, 2 weeks, 3 weeks, and 4 weeks after intervention were lower compared to the control group (*P* < 0.05). The comparison of social support showed that the scores of objective support, subjective support, utilization of support, and total score of social support in the study group were higher compared to the control group (*P* < 0.05). The number of abortions in the control group was lower compared to the control group, and the number of full-term deliveries was higher compared to the control group (*P* < 0.05). Finally, we compared the scores of life quality. After nursing, the scores of life quality of the two groups increased. Of note, the scores of physiological function, psychological function, social function, and health self-cognition in the study group were lower compared to the control group (*P* < 0.05).

RETRACTED

**Conclusion:**

Comprehensive nursing for patients with APS based on Orem's self-care theory can effectively improve clinical symptoms and pregnancy outcome and play a positive role in facilitating patients' nursing satisfaction and self-nursing ability, which can also effectively strengthen mental health and social support, this nursing model is worth popularizing in clinic.

## 1. Introduction

Antiphospholipid syndrome (APS) is a noninflammatory autoimmune disease characterized by persistent high titer positive antiphospholipid antibodies (APL) [1]. The most common clinical manifestations are arterial or venous thrombosis and/or recurrent bad pregnancy. The common APL that are significant for the diagnosis of APS are anticardiolipin antibodies (ACL), anti-*β* 2-glycoprotein I (*β*-2GPI) antibodies, and lupus anticoagulant (LA) antibodies. APS is more common in young women of childbearing age. Women account for about 70% of APS patients, and the incidence is the highest during pregnancy [2]. Some studies have indicated that APL is a risk factor for thrombosis. If the three antibodies (ACL, LA, anti-*β* 2-GP I antibody) in patients with APS are all positive, the risk of thrombosis increases [3]. Recurrent abortion refers to the abortion that occurs more than 2 times with the same partner and occurs before 20 weeks of pregnancy, which is an important reason of female infertility. The most common obstetrical complication of APS is abnormal pregnancy, most of which are recurrent abortion, and about 80% of the patients are early pregnancy (before 12 weeks of pregnancy) abortion [4]. According to the literature, the probability of pregnancy loss in APS patients is from 23.8% to 52.3%, and recurrent abortion and fetal death are the most common in uterus; about 5%-20% of recurrent abortion patients have persistent antiphospholipid antibody positive; if there is no clinical intervention, up to 90% of antiphospholipid antibody positive patients can have unsuccessful pregnancy again [5]. Therefore, strengthening the understanding of pregnancy complicated with APS is conducive to better clinical intervention, reduce the incidence of thrombosis and pregnancy complications, and improve the pregnancy outcome of patients [6].

Orem's self-care theory was originally put forward by Dorothea Orem, an American nursing theorist [7]. Self-care is an individual's self-care behavior and activities to meet the maintenance of their own life, health function, growth, development, and happiness, which is realized by meeting the existing self-care needs [8]. In recent years, there have been more investigations and applications on self-care behavior, which have developed rapidly, mainly focused on chronic diseases such as chronic obstructive pulmonary disease, asthma, heart failure, diabetes, hypertension, and hemiplegia [9]. The results indicate that after self-nursing intervention, patients can master the relevant knowledge of the disease, correctly understand the disease and self-worth, and adapt to various changes caused by illness [9]. Active participation in the treatment and rehabilitation of the disease can enhance the quality of life of patients. Orem's self-care theory emphasizes the individual's self-care ability, which is consistent with the nursing concept of “patient-centered” holistic nursing [10]. Its purpose is to strengthen personal health and the physical coping skills of the body and has gradually become the main means of chronic diseases management [11]. Comprehensive nursing is a nursing model that integrates psychological nursing, diet intervention, health education, and other nursing methods. This nursing strategy pays more attention to the comprehensiveness and integrity of nursing methods, while the comprehensive nursing based on Orem's self-care theory is guided by Orem's self-care theory and carries out comprehensive nursing according to Orem's self-care theory, which can take targeted nursing intervention measures for patients more effectively [12].

RETRACTED

APS has a serious impact on people's lives and health [13]. In order to promote the life quality of patients with APS, it is imperative to facilitate the self-care ability of patients with APS. In line with the current requirements of high-quality nursing services, patients' self-care ability has been improved in order to return more time to nurses, and nurses can more efficiently spend their time on patients who really need it. Meanwhile, with the innovation and progress of medical technology in recent years, the number of patients with APS is also increasing, in order to strengthen the life quality of patients after discharge and reduce the burden of society and families. It is also very valuable to promote the self-care ability of patients [13, 14]. In the process of self-nursing intervention, the most important thing is to completely change the mind that patients are dependent on medical staff and their families, make them consciously realize the importance and significance of self-care ability, and constantly mobilize patients' enthusiasm and sense of participation; make patients from simple passive treatment and nursing to actively participate in treatment and nursing activities, gradually assume the responsibility of self-care [13]. In the past, routine nursing was adopted for patients with APS, but the nursing effect was not satisfactory. Based on this, this study focuses on the effect of comprehensive nursing based on Orem's self-care theory on the improvement of symptoms and pregnancy outcome of patients with APS. The results are reported as follows.

RETRACTED

## 2. Patients and Methods

### 2.1. General Information

Sixty patients with APS treated in our hospital from February 2019 to April 2021 were enrolled. The control group received routine nursing, and the study group received comprehensive nursing based on Orem's self-care theory. In the control group, the age was 21-44 years old, the average age was 32.94 ± 3.63 years old. In the study group, the age was 20-45 years old, the average age was 32.931 ± 3.66 years old. There was no statistical significance in the general data of the two groups. This study was permitted by the Medical Ethics Association of our hospital and all patients noticed informed consent.

Inclusion criteria are as follows: (1) age ≥ 18 years old; (2) no cognitive, language and intellectual impairment, basic reading and writing ability; and (3) consent to follow-up for 6 months and be able to accept and answer telephone followers.

Exclusion criteria are as follows: patients with SLE, hematopathy, heart disease, genetic disease, hyperthyroidism, hypothyroidism, and other diseases that can lead to abortion or thrombosis and incomplete data were excluded.

### 2.2. Treatment Methods

The control group received comprehensive nursing, issued disease guidance manuals to patients on the day of admission, evaluated admission, patiently carried out health education for patients, explained to patients matters needing attention in disease-related self-management, and gave individualized nursing guidance. Education is mainly carried out through health education.

Compared to the control group, the study group carried out comprehensive nursing based on Orem's self-care theory. The specific measures are as follows: (1) complete compensation system: at this stage, patients are unable to take care of themselves and have a low level of self-care ability. Due to adverse pregnancy outcomes, patients have no time to take care of themselves at this time the use of complete compensation system to compensate for patients' lack of self-care. Meanwhile, the patients are in a negative mood and need to be comforted by others. To relieve the patients' emotions, nurses should strengthen their communication with patients, understand the types of music they like, and choose relaxing and decompression music according to their wishes, such as “brook chanting” and “sea reverie.” Guide patients to follow the music rhythm for progressive muscle relaxation. Tighten the hands, forearms, upper arms, forehead, cheeks, nose, lower jaw, shoulder and neck, chest and back, abdomen, thighs, calves, and feet in turn, and relax after holding for (5-7) seconds. And 30 min/times, once a day; (2) partial compensation system: at this stage, the level of patients' self-care ability is moderate, some of them need nurses to provide nursing care, and both nurses and patients play a certain role in satisfying self-care. Then, nurses provide partial compensatory care to mobilize patient initiative. Next, nurses should be considerate and care for patients, enumerate cure cases, encourage patients to speak for themselves, and encourage family members to accompany and care, so as to establish the belief that patients can restore their health. In addition, nurses should also enhance image guidance on the basis of the original music relaxation training, that is, under the background music, they should instruct patients to carry out progressive muscle relaxation while imagining a happy life experience under the guidance of instructions; (3) support-education system: at this stage, the level of self-care ability of patients is at a high level, which belongs to the type of mild dependence. Patients have the ability to implement or learn some necessary self-care methods, but they must consult a nurse and complete it under the guidance and education: (1) provide psychological care to family members and seek emotional support from family members. Improve communication with the patient's family and inform them that venting anger is a normal psychological process for the patient. In addition, they should also explain the simple psychological nursing knowledge (such as listening, persuasion, comfort, and appropriate physical contact). Encourage family members to visit and accompany; (2) to guide the patients to vent their emotions reasonably. Patients are encouraged to vent their anger by writing diaries, pouring out your feelings, listening to music, sports, and other ways. In addition, nurses should care and understand patients and analyze irrational concepts in view of patients in order to correct their misunderstandings.

RETRACTED

### 2.3. Observation Index

#### 2.3.1. Satisfaction

After consulting the literature and expert discussion, we designed patients' follow-up satisfaction, a total of 10 items, and recorded patients' satisfaction with follow-up management mode, health education, medical and nursing service, appointment registration process, and so on [14]. It is divided into four dimensions: very satisfied, satisfied, general, and dissatisfied. Satisfaction rate = very satisfaction rate + satisfaction rate + general rate.

#### 2.3.2. Self-Care Ability

Self-care ability scale (ESCA): the scale was designed according to Orem's self-care theory [15]. Invented by Kearny and Fleisher in 1979, it is used to investigate the patients' self-care ability. There are 4 dimensions and 43 items: self-concept, sense of self-care responsibility, self-care skills, and health knowledge [16]. The score of each item of the scale was 0-4, of which 11 were reverse scores, with a total score of 172. According to the total score of the scale and the score of each item, the self-nursing ability was divided into three levels: <33% of the total score was low level, 33% to 66% of total score was medium level, >66% of total score was high level, and the higher the score was.

#### 2.3.3. Self-Rating Anxiety Scale (SAS)

Compiled by Zung in 1971, it was used to evaluate the subjective feelings of anxiety patients. There were 20 questions, containing 4 reverse scores [16]. The answers were divided into 4 grades and the positive scores were 1, 2, 3, and 4, respectively. The reverse score is 4, 3, 2, and 1, respectively. The total scores for the 20 themes were added together to obtain the total score. In the scale cooperation group, 1158 Chinese normal subjects were studied. The results indicated that the average gross score was 29.78 ± 10.07, and the normal upper limit of the total gross score was 40 points.

#### 2.3.4. Social Support Rating Scale (SSRS)

Compiled by Xiao Shuiyuan in 1986 and tested by a large sample of people in the community, it is proved to have good reliability and validity, and it is widely employed in the field of psychosomatic medicine in China [17]. The scale includes three dimensions: objective support (3 items), subjective support (4 items), and utilization of social support (3 items). There are 10 items in the scale, only 1 item is enrolled for each item of item 1-4 and item 8-10, and items 1, 2, 3, and 4 are enrolled, and the scores are 1, 2, 3, and 4, respectively. Article 5 is divided into items A, B, C, D, and E5, score 0-4 for each item from zero to full support; Articles 6 and 7, if you answer “there is no source”, score 0. If you answer “the following sources,” you will get a few points from several sources. The total score is the sum of 10 items. The total score ranges from 12 points to 66 points, the higher the score, the higher the social support, lower than 33 points as low social support, 33 to 45 points as average social support, and higher than 45 points as high social support.

#### 2.3.5. Pregnancy Outcome

The pregnancy outcomes of the two groups were calculated. Containing: miscarriage, stillbirth, premature delivery, and full-term delivery.

#### 2.3.6. Life Quality Scale

The scale of life quality consists of four subscales, containing physical, psychological, social, and health self-awareness with a total of 29 items. Cronbach's *α* coefficient of the scale is 0.79 to 0.91. The scale was scored by 1-5 grades. The lower the score, the higher the satisfaction.

RETRACTED

### 2.4. Statistical Analysis

The obtained data were analyzed by using SPSS Statistics 22.0 software. The measurement data were tested by normality test and variance homogeneity test. The normal distribution was presented by mean ± standard deviation (*x* ± *s*), compared with *t*-test, the nonnormal distribution was presented by median and quartile *M* (Q1 ~ Q3), and the rank sum test was employed for comparison. Counting data line chi-square test. The above test, *P* < 0.05 indicates that the difference is statistically significant.

## 3. Results

### 3.1. Comparison of Nursing Satisfaction

First of all, we compared the nursing satisfaction. The study group was very satisfied in 23 cases, satisfactory in 5 cases, and general in 2 cases, and the satisfaction rate was 100%. The control group was very satisfied in 11 cases, satisfactory in 10 cases, general in 4 cases, and dissatisfied in 5 cases. The satisfaction rate was 83.33%. The nursing satisfaction in the study group was higher compared to the control group (*P* < 0.05). All the data results are indicated in Figure 1.

### 3.2. Comparison of Self-Nursing Ability Score

Secondly, we compared the score of self-nursing ability. The self-concept, sense of self-care responsibility, self-nursing skills, health knowledge, and total score of the study group were higher compared to the control group (*P* < 0.05). All the data results are indicated in Table 1.

### 3.3. Anxiety Score Comparison

Thirdly, the anxiety scores of the two groups were compared. Before intervention, there exhibited no significant difference (*P* > 0.05). The anxiety scores of the study group before intervention, 1 week, 2 weeks, 3 weeks, and 4 weeks after intervention were lower compared to the control group (*P* < 0.05). The results of all the data are indicated in Table 2.

### 3.4. Comparison of Social Support

Then, we compared the status of social support. The study group objective support, subjective support, support utilization, and the total score of social support were higher compared to the control group (*P* < 0.05). All the data results are indicated in Table 3.

### 3.5. Comparison of Pregnancy Outcome

There were 5 cases of abortion, 2 cases of stillbirth, 2 cases of premature delivery, and 21 cases of full-term delivery in the study group, while 7 cases of abortion, 2 cases of stillbirth, 10 cases of premature delivery, and 11 cases of full-term delivery in the control group. The number of abortions in the study group was lower compared to the control group, and the number of full-term deliveries in the study group was higher compared to the control group (*P* < 0.05). All the data results are indicated in Figure 2.

RETRACTED

### 3.6. Comparison of Qualities of Life Scores

There exhibited no significant difference in the score of quality of life before nursing (*P* > 0.05). The scores of physiological function, psychological function, social function, and health self-cognition in the study group were lower compared to the control group (*P* < 0.05). All the data results are indicated in Table 4.

## 4. Discussion

The effect of APS on abortion has been paid attention to by obstetricians and gynecologists [18]. Women of childbearing age with this will have an increased risk of recurrent abortion or other obstetrical complications. APL include ACL and LAs, which can cause placental vascular thrombosis, placental infarction, and placental dysfunction [19]. Other studies have suggested that it may inhibit trophoblast cell erosion and differentiation and lead to early abortion [20]. Anticoagulant therapy, glucocorticoid, and immunotherapy have been widely employed in clinic for recurrent abortion caused by APS, and aspirin has become a routine treatment. According to the revised standard of Sapporo in 2006, the laboratory standard of APS is that medium and high titers of IgG or IgM ACL or LAs or *β* 2GPI antibodies were found in at least 2 or more examinations at intervals of 6 weeks. In addition to laboratory diagnosis, clinical diagnosis is also very important. Many obstetrical complications related to APS have been proposed in the newly revised diagnostic criteria of APS. However, the diagnosis and treatment of APS are still controversial. The understanding of the etiology and pathogenesis of APS is still limited. APS is now widely considered to be a coagulation disorder, so heparin or aspirin is often applied for anticoagulation. However, recent studies on the animal model of APS suggest that the etiology of obstetrical complications caused by APS is mainly mediated by inflammation, not thrombosis. The study suggests that anti-inflammatory therapy should be employed in the treatment of APS. Meanwhile, these studies have also discussed that the potential mechanism of recurrent miscarriage as possibly being muscle damage caused by APL expression. Heparin can inhibit this pathogenic factor and is effective in the treatment of APS obstetrical diseases [21].

APL are a series of autoimmune antibodies, the existence of which is related to thrombosis and recurrent abortion [22]. Regardless of the titer of anticardiolipin antibody, anticardiolipin antibody can bind to phospholipids on plasma proteins, such as prothrombin, *β*-2GPI, and V-annexin, and become a risk factor for thrombosis in patients with systemic lupus erythematosus or recurrent abortion [23]. These antibodies are more common and have higher titers in patients with primary APS and systemic lupus erythematosus than in patients with recurrent abortion. APL IgG or IgM, anti-*β* 2GPI antibodies, anti-PT antibodies, and anti-V annexin antibodies accounted for 100%, 80%, 60%, and 24% of primary APS patients, respectively, compared with 66% of recurrent abortion patients whose above antibodies were negative, of which ACL IgG or IgM, anti-*β* 2GPI antibodies, anti-PT antibodies, and anti-V annexin antibodies accounted for 6%, 6%, 16%, and 17%, respectively [23]. Thrombosis and thrombocytopenia are common in patients with SLE and primary APS, but rare in patients with recurrent abortion. One study indicated that the APL of pregnant women with a history of recurrent abortion was higher compared to normal pregnant women [24]. The detections of ACL and anionic phospholipid antibodies in 320 patients with recurrent abortion indicated that antibody titers have reached moderate levels, some of which are even at high levels, while others are negative. When these patients were treated with heparin or aspirin, 64% responded to treatment and could have a normal pregnancy. Obstetrical APS is defined as the complications of pregnancy, such as recurrent abortion, stillbirth, preterm delivery, severe preeclampsia, and postpartum hemorrhage. The laboratory index is confirmed as APS [25]. Among them, HELLP syndrome may be related to antiphospholipid microvascular lesions and microvascular hemolysis. For patients with APA-positive recurrent abortion, the pathological changes of microvascular thrombosis and microvascular hemolysis in placenta are still unknown, and more investigations are needed in the future.

RETRACTED

There are several mechanisms to explain the clinical manifestations associated with APL: (1) first, APL can activate platelets, endothelial cells, and monocytes, leading to thrombosis and thrombocytopenia, which is also a common complication of APS [26]. We can speculate that platelet activation may be the most important part of APL-mediated immunopathology. APL can increase the expression of glycoproteins on platelet membrane, especially GPIIb/IIIa and GPIIIa [27]. There is also sufficient evidence to indicate that APL can activate endothelial cells and monocytes, resulting in increased expression of different cell adhesion molecules and tissue factors. ACL-induced thrombosis was also related to the titer of ACL, but not to the titer of phospholipid antibodies with anions [26, 27]. In an animal experiment, leukocyte adhesion to endothelial cells induced by ACL also reflected a concentration-dependent effect [28]; (2) APL-induced placental and vascular bed thrombosis is caused by interfering with the anticoagulant effect of Annexin A5 on the surface of phospholipids. The aggregation of Annexin A5 on the surface of phospholipids leads to the translocation of coagulation factor Va and prevents the formation of procoagulant complexes. Decidual artery thrombosis was found by histological analysis, but there was not enough evidence to indicate inflammatory cell infiltration in decidua and fetal tissue. In this case, abortion is related to the procoagulant activity of CICI5, not because of the intervention of Annexin A5, because CICI5 cannot destroy the normal sequence distance between Annexin A5 [28, 29]. Therefore, there are many ways to induce placental and vascular bed thrombosis mediated by APL. (3) APL can change the maturation, differentiation, and erosion of trophoblasts. Histopathological examination indicated that abortion in APA-positive pregnant women during 7-10 weeks of pregnancy was mainly due to intravascular trophoblast erosion of decidual vessels without excessive chorionic thrombosis. This finding suggests that APL causes placental dysfunction, and thrombosis is not the only explanation for obstetrical complications in patients with APS [25]. It has been proved that anti-*β* 2GPI antibody can trigger the inflammatory response in trophoblast cells by increasing the secretion of IL-8, MCP-1, GRO-*α,* and IL-1 *β*. When the concentration is high, these antibodies can cause caspase-mediated apoptosis [26]. Therefore, by acting on autocrine and paracrine, *β* 2GPI antibody will induce inflammatory mediators to destroy trophoblast cells. In addition, APL can restrict trophoblast migration by downregulating the secretion of IL-6 and reducing the activity of STAT3 in trophoblast cells [27]. Therefore, women with APL and recurrent abortion have an increased risk of obstetrical complications. APL can reduce the products of VEGF and MMPs and the NF-*κ*B DNA binding activity at the molecular level. After recognizing phospholipids with anions and *β*-2GPI, APL can adhere to trophoblast cells, which can reduce the release of *β*-hCG and erosion of basement membrane. Therefore, APL can destroy the maturation, movement, and erosion of trophoblast cells.

The theory of Orem's self-care was put forward by the famous American nursing scientist Orem (Dorothea. E. Orem) in her book Nursing: Concepts of Practice. Self-care theory holds that self-care is a behavior created and taken by human individuals to survive, maintain, and promote health and tranquility and emphasizes that the ultimate goal of nursing is to restore and enhance the self-care ability of individuals, families, and even the whole society [28]. Orem's self-care defect theory divides the nursing procedure into three steps: diagnosis and treatment, design and planning implementation, and evaluation. Some scholars have pointed out that the self-care theory is not only applicable to patients but also to the study of caregivers. Self-care theory emphasizes self-care as the center, and the ultimate goal is to make individuals bear the responsibility of self-care. It includes five aspects: the behavior of self-care, the ability of self-care, the need of therapeutic self-care, the basic elements that affect the individual's demand for therapeutic self-care and self-care ability, and the constituent elements of individual ability to complete self-care activities [29]. Self-care defect theory is the core of Orem's self-care model, in order to meet patients' self-care defects or deficiencies and then facilitate the overall self-care ability of patients. When the lack of self-care ability cannot meet the needs of therapeutic self-care, there will be self-care defects, which require nurses to provide professional care to compensate for self-care defects. Three kinds of dynamic and continuous nursing systems, namely, full compensation system, partial compensation system, and support-education system, constitute the theory of nursing system [30]. Its function is that when the patients' therapeutic self-care needs cannot be met, both nurses and patients need to undertake and implement the corresponding nursing contents and nursing measures. Meanwhile, it is pointed out that medical staff should adopt different nursing systems according to patients' different self-care ability and needs. When a patient is completely unable to carry out self-care due to the limitation of his illness or other factors, it is necessary for nurses to employ the full compensation system to give comprehensive nursing on the basis of evaluating their self-care needs, but the patient's self-care ability should be evaluated timely and dynamically to avoid providing excessive compensation help, resulting in overdependence of patients [31]. When patients can complete self-care in some aspects but have insufficient self-care, it is necessary for nurses to employ part of the compensation system to make up for the deficiency of their self-care ability. At this time, patients should be actively guided to participate in their own health management, give patients more opportunities for self-care, give timely encouragement to patients' progress, and enhance patients' confidence and sense of achievement in self-care. When patients are lack of self-care knowledge and have the ability to learn how to self-care, nurses need to employ the support-education system to provide psychological and technical guidance and support to improve their self-care ability. Concomitantly, provide as much disease-related knowledge and self-nursing skills as possible, and teach patients to apply to their own diseases [30, 31]. We should make comprehensive use of these three systems from a developmental and open viewpoint, which cannot be applied in isolation or completely separated and used.

RETRACTED

The main purpose of self-care is to make patients less dependent on others and to make patients realize that the work of medical staff can only help them to recover from treatment, but cannot be completely replaced [32]. In the process of self-nursing intervention, weakening the role of patients, patients' families or medical staff should avoid providing excessive complete compensation system to patients, avoid overdependence of patients, and fully give patients the opportunity to exercise themselves, help them build up self-confidence in overcoming the disease, constantly mobilize patients' enthusiasm and participation consciousness, and make patients actively participate in treatment and nursing activities [31, 32]. The self-care needs of patients are different in various treatment stages of the disease. When the self-care model is applied to the nursing of head cancer patients, patients are personally involved in their own health decision-making and management during hospitalization. So that patients have a deeper understanding of the treatment and nursing activities received during hospitalization, and then better cooperate with the treatment and promote the rehabilitation of patients. The continuous comprehensive nursing program for patients with antiphospholipid syndrome based on Orem's self-care theory, through cognitive behavioral therapy and psychological staging support therapy, according to the patient's personality characteristics and educational level, takes the patient as the must, takes the family as the unit, carries on the step-by-step and reasonable nursing plan to the patient's disease, corrects the patient's wrong cognition and behavior, and helps correct the patient's distorted cognitive model [32, 33]. With the extension of comprehensive nursing, the depression score of patients with APS decreased significantly after nursing, which was significantly lower compared to before nursing. This indicates that comprehensive nursing based on Orem's self-care theory is better than conventional nursing in the rehabilitation process of patients with APS. And some problems encountered after discharge can also be solved; meanwhile, comprehensive nursing can be strengthened again. This is consistent with the results on the value of comprehensive psychological nursing for patients with postoperative depression after APS [33]. According to the different psychological problems of the patients, support, attention, and guidance were given from different aspects to reduce the degree of depression of the patients, which promotes mental health, strengthens the psychology of medical compliance, and improves the prognosis and quality of life of patients with APS. Psychological nursing is very suitable for patients with APS in the early stage where various treatments are relatively concentrated. Therefore, comprehensive nursing can effectively enhance the depression state of patients with APS and facilitate their quality of life.

RETRACTED

Conclusively, comprehensive nursing for patients with antiphospholipid antibody syndrome based on Orem's self-care theory can effectively promote clinical symptoms and pregnancy outcome and play a positive role in facilitating patients' nursing satisfaction and self-nursing ability, which can also effectively strengthen mental health and social support, this nursing model is worth popularizing in clinic.

## Figures and Tables

**Figure 1:** Comparison of patient satisfaction between two groups. The green bar represents the control group and the yellow bar represents the research group.

**Figure 2:** Comparison of pregnancy outcomes between two groups. The green bar represents the control group and the yellow bar represents the research group.

**Table 1:** Comparison of self-nursing ability scores between the two groups [$\bar{x}\pm s$, Points].

Group	*N*	Self-concept	Sense of responsibility for self-care	Self-nursing skills	Health knowledge level	Total score
C group	30	14.31 ± 3.16	15.66 ± 3.31	17.59 ± 3.12	23.28 ± 2.21	70.85 ± 2.14
R group	30	18.93 ± 6.42	17.49 ± 1.56	20.58 ± 2.12	30.68 ± 3.31	85.81 ± 1.23
*t*		3.530	2.739	4.341	10.183	33.196
*P*		<0.01	<0.01	<0.01	<0.01	<0.01

**Table 2:** Comparison of anxiety scores between the two groups [$\bar{x}\pm s$, Points].

Group	*N*	Before intervention	One week after intervention	2 weeks after intervention	3 weeks after intervention	4 weeks after intervention
C group	30	56.38 ± 1.18	53.12 ± 3.55	48.64 ± 2.44	44.42 ± 1.11	40.42 ± 1.42
R group	30	56.82 ± 1.64	45.31 ± 3.34	42.44 ± 2.65	40.66 ± 3.54	36.77 ± 1.44
*t*		1.192	8.776	9.427	5.551	9.885
*P*		>0.05	<0.01	<0.01	<0.01	<0.01

**Table 3:** Comparison of social support between the two groups [$\bar{x}\pm s$, Points].

Group	*N*	Objective support	Subjective support	Support utilization	Total score of social support
C group	30	8.21 ± 0.41	23.42 ± 1.56	7.42 ± 0.56	37.13 ± 2.65
R group	30	9.99 ± 0.53	25.33 ± 1.42	8.56 ± 0.55	42.77 ± 0.14
*t*		14.549	4.959	7.954	11.640
*P*		<0.01	<0.01	<0.01	<0.01

RETRACTED

**Table 4:** Comparison of life quality scores between the two groups before treatment [$\bar{x}\pm s$, Points].

Group	*N*	Physiological function		Psychological function		Social function		Healthy self-cognition	
		Before nursing	After nursing	Before nursing	After nursing	Before nursing	After nursing	Before nursing	After Nursing
C Group	30	15.84 ± 4.91	13.86 ± 2.95^a^	16.94 ± 3.91	14.85 ± 4.86^a^	18.82 ± 3.95	16.37 ± 2.81^a^	15.98 ± 3.91	13.86 ± 1.85^a^
R Group	30	15.96 ± 4.52	11.84 ± 2.91^b^	16.95 ± 3.86	12.81 ± 1.85^b^	18.84 ± 3.55	12.84 ± 3.81^b^	15.87 ± 3.66	10.83 ± 2.91^b^
*t*		0.098	2.670	0.009	2.148	0.020	4.084	0.112	4.812
*P*		0.921	0.009	0.992	0.035	0.983	0.000	0.910	0.000

Note: the control group before and after nursing, ^a^*P* < 0.05; the study group before and after nursing, ^b^*P* < 0.05.

## Data Availability

No data were used to support this study.
